# LncRNA TCF7 Promotes Epithelial Ovarian Cancer Viability, Mobility and Stemness *via* Regulating ITGB8

**DOI:** 10.3389/fonc.2021.649655

**Published:** 2021-11-17

**Authors:** Changlei Su, Kejin Huang

**Affiliations:** ^1^ Department of General Surgery, The Second Hospital of Harbin Medical University, Harbin, China; ^2^ Department of Gynecology, Harbin Medical University Cancer Hospital, Harbin, China

**Keywords:** long non-coding RNAs T-cell factor 7, epithelial ovarian cancer, clinicopathological features, overall survival, integrin β8, cancer stem cells

## Abstract

This study aimed to investigate the carcinogenic role of long non-coding RNA T-cell factor 7 (lnc-TCF7) in epithelial ovarian cancer (EOC). Lnc-TCF7 overexpression and shRNA plasmids were transfected into SKOV3 and OVCAR3 cells, followed by measurement of cell proliferation, migration, invasion, apoptosis, stemness, and mRNA profile (via microarray). Besides, lnc-TCF7 expression was measured in tumor and adjacent tissues from 76 EOC patients. Lnc-TCF7 was upregulated in EOC cell lines; its overexpression increased cell proliferation, migration, invasion, but decreased apoptosis and promoted CD44, CD133 expressions, CD44^+^CD133^+^ cell proportion, spheres formation efficiency and drug resistance to cisplatin in SKOV3 and OVCAR3 cells. Besides, lnc-TCF7 ShRNA exhibited opposite effects comparing with its overexpression. Microarray analysis revealed 267 mRNAs were modulated by lnc-TCF7 dysregulation, among which ITGB8 was the most dysregulated one, which was validated by subsequent western blot and RT-qPCR. Furthermore, ITGB8 overexpression not only induced proliferation, migration, invasion and stemness, but also attenuated the effect of lnc-TCF7 ShRNA on these functions in SKOV3 and OVCAR3 cells. In addition, lnc-TCF7 was upregulated in tumor tissues and correlated with higher pathological grade, tumor size, International Federation of Gynecology and Obstetrics (FIGO) stage and worse overall survival in EOC patients. Conclusively, lnc-TCF7 regulates multiple oncogenic pathways, promotes proliferation, migration, invasion, stemness *via* upregulating ITGB8. It also correlates with advanced tumor features and poor prognosis in EOC, implying its potential as a target for EOC treatment.

## Introduction

Epithelial ovarian cancer (EOC) is the most lethal malignancy of the female reproductive tract, which accounts for 5% of all cancer cases. EOC is also the seventh most frequent malignant neoplasm and the eighth most common cause of cancer-associated mortalities with approximately 4.2% mortality rate among females worldwide (1–3). With the development of various treatment modalities for EOC, including surgical resection, chemotherapy, radiotherapy, targeted therapy and immunotherapy (4), EOC patients could realize a satisfactory prognosis if diagnosed at the early stage of the disease. However, nearly 70% of EOC patients are diagnosed at an advanced stage [International Federation of Gynecology and Obstetrics (FIGO) stage III or IV] due to non-specific symptoms. Besides, the 5-year survival rate of patients with EOC is less than 30% (4). Therefore, a deeper understanding of the molecular mechanisms underlying EOC progression is required to develop novel therapeutic agents and improve patient outcomes.

Long non-coding RNA (lncRNA), a class of non-coding RNA, possesses a length of more than 200 nucleotides and lacks protein-coding ability. It commonly locates within intergenic stretches or overlapping antisense transcripts of protein-coding genes. lncRNAs are involved in regulating several biological processes, including cell proliferation, apoptosis, migration, invasion and differentiation (5). Accumulating evidence suggests that lncRNAs may play important roles in tumorigenesis and tumor progression (6). Among previously reported lncRNAs, lncRNA T-cell factor 7 (lnc-TCF7) serves as a vital oncogene, which contributes to malignant behaviors and cancer stemness in several carcinomas, such as non-small cell lung, colorectal and liver cancers (7–10). Besides, lnc-TCF7 exhibits potency as a prognostic marker reflecting advanced tumor stages and worse survival in some carcinomas (11–13). However, no previous studies have been performed on the function and mechanism of lnc-TCF7 in EOC, as well as its clinical value for EOC prognosis.

Our preliminary study revealed that lnc-TCF7 was upregulated in EOC cell lines and tissues. Consequently, the present study explored the function and molecular mechanisms of lnc-TCF7 in EOC. Specifically, the present study examined the roles of lnc-TCF7 in EOC cell proliferation, apoptosis, migration, invasion, stemness; meanwhile, this study explored the EOC-associated regulatory network and target genes of lnc-TCF7. Furthermore, the association of lnc-TCF7 with clinicopathological features and overall survival (OS) in patients with EOC was investigated.

## Materials and Methods

### EOC Cell Culture and lnc-TCF7 Expression

The EOC cell lines CAOV3 (ovarian serous adenocarcinoma), SKOV3 (ovarian serous cystadenocarcinoma) and OVCAR3 (ovarian serous adenocarcinoma) were purchased from the Cell Bank of Chinese Academy of Sciences. The EOC cell line UWB1.289 (ovarian carcinoma) was purchased from the American Type Culture Collection. The normal ovarian epithelial cell line IOSE80 was purchased from BioVector NTCC Inc. SKOV3, OVCAR3, UWB1.289 and IOSE80 cells were cultured in 90% Roswell Park Memorial Institute Medium (RPMI)-1640 (Gibco; Thermo Fisher Scientific, Inc.) supplemented with 10% fetal bovine serum (FSB; Gibco; Thermo Fisher Scientific, Inc.) at 37°C in a humidified atmosphere containing 5% CO_2_. CAOV3 cells were cultured in 90% DMEM (Gibco, USA) supplemented with 10% FBS at 37°C in a humidified atmosphere containing 5% CO_2_. Lnc-TCF7 expression in CAOV3, SKOV3, OVCAR3, UWB1.289 and IOSE80 cells was detected by reverse transcription-quantitative polymerase chain reaction (RT-qPCR).

### Effect of lnc-TCF7 Dysregulation on EOC Cell Functions

Lnc-TCF7 overexpression and negative control (NC) overexpression plasmids were constructed using pEX-2 vector, while lnc-TCF7 knockdown and NC knockdown shRNAs were constructed using pGPU6 plasmids (Shanghai GenePharma Co., Ltd., China). Then they were transfected into SKOV3 and OVCAR3 cells using HilyMax (Dojindo Molecular Technologies, Inc.) and OPTI-MEM (Thermo Fisher Scientific, Inc.), which named as OE-NC, OE-TCF7, SH-NC, SH-TCF7, respectively. Following that, lnc-TCF7 expression, proliferation, apoptosis, apoptotic markers, migration, invasion, CD44 expression, CD133 expression, CD44^+^CD133^+^ cell proportion, sphere formation ability, cisplatin sensitivity were detected. It was worthy noticing that shRNA was used in our study but not siRNA, since Sphere Formation Assay needed longer lasting effect of knockdown which shRNA achieved better (14).

### Microarray and Bioinformatics Analyses

SKOV3 cells (5x10^6^) from OE-NC vs. OE-TCF7, SH-NC vs. SH-TCF7 groups were harvested at 24 h post transfection, then the total RNA was extracted using TRIzol reagent (Invitrogen; Thermo Fisher Scientific, Inc.). The quality of the extracted RNA was assessed by the NanoDrop ND-2000 spectrophotometer (Thermo Fisher Scientific, Inc.). Then the RNA was proposed to gene expression profiling applying Agilent 4 x 44 Kv2 expression arrays (Agilent Technologies, Inc.) by a third company (Jinneng Bio-Tech Co., Ltd.). After the data processing conducted by the third company, raw data was analyzed using R software (version 3.3.3, https://www.r-project.org/). Differentially expressed genes (DEGs) were identified using the limma package (version 3.6.9, http://bioconductor.org/packages/2.7/bioc/html/limma.html). P<0.05 and a fold-change (FC) >1.5 were considered to indicate a statistically significant difference. The DEGs heatmap was constructed through the usage of the pheatmap package (version 1.0.12, https://mirrors.tongji.edu.cn/CRAN/). Gene Ontology (GO) and Kyoto Encyclopedia of Genes and Genomes (KEGG) enrichment analyses of the DEGs were performed by application of the Database for Annotation, Visualization and Integrated Discovery.

Furthermore, cross-analysis to identify the overlapping DEGs between the OE-TCF7 vs. OE-NC groups, between the SH-TCF7 vs. SH-NC groups was performed. DEGs that were upregulated in the OE-TCF7 (vs. OE-NC) group and downregulated in the SH-TCF7 (vs. SH-NC) group, or downregulated in the OE-TCF7 (vs. OE-NC) group and upregulated in the SH-TCF7 (vs. SH-NC) group were selected as accordant DEGs for subsequent heatmap construction as well as GO and KEGG enrichment analyses.

Top 5 according genes [sorting nexin 2 (SNX2), protocadherin β-8 (PCDHB8), integrin β8 (ITGB8), interleukin 1 α (IL-1A) and fibronectin (FN1)] were chosen as candidate targets of lnc-TCF7, by the rank by the sum of absolute value of Log_2_FC[OE-TCF7/OE-NC] and Log_2_FC[SH-TCF7/SH-NC]. All of them were further validated by western blot and RT-qPCR, respectively.

### ITGB8 Dysregulation on EOC Cell Proliferation, Apoptosis, Migration, Invasion, Stemness and Cisplatin Sensitivity

NC knockdown, lnc-TCF7 knockdown, NC overexpression, ITGB8 overexpression plasmids were transfected into SKOV3 cells alone or in combination with HilyMax and OPTI-MEM, which were named as SH-NC + OE-NC, SH-NC + OE-ITGB8, SH-TCF7 + OE-NC, SH-TCF7 + OE-ITGB8, respectively.

Besides, NC overexpression, lnc-TCF7 overexpression, NC knockdown, ITGB8 knockdown were transfected into OVCAR3 cells alone or in combination with the use of HilyMax and OPTI-MEM, which were named as SH-NC + OE-NC, SH-NC + OE-ITGB8, SH-TCF7 + OE-NC, SH-TCF7 + OE-ITGB8, respectively.

Following that, lnc-TCF7 expression, ITGB8 expression, proliferation, apoptosis, apoptotic markers, migration, invasion, CD44 expression, CD133 expression, CD44^+^CD133^+^ cell proportion, sphere formation ability, cisplatin sensitivity were detected.

### Western Blotting

Total protein was extracted and a bicinchoninic acid kit (Pierce; Thermo Fisher Scientific, Inc.) was used to measure the protein concentration. Total protein (20 μg/lane) was separated *via* SDS-PAGE on a 10% gel and transferred onto a polyvinylidene fluoride membrane (EMD Millipore). The membrane was blocked by incubating with 5% skim milk for 2 h. The membrane was incubated with the primary antibodies (**Supplementary Table 1**) overnight at 4°C. Following primary antibody incubation, the membrane was incubated with secondary antibodies (**Supplementary Table 1**) for 1 h at room temperature. The protein bands were visualized using an enhanced chemiluminescence kit (EMD Millipore). GAPDH served as the loading control.

### RT-qPCR

Cells were digested using 0.25% trypsin (Gibco; Thermo Fisher Scientific, Inc.) and collected. Total RNA was extracted using TRIzol reagent (Invitrogen; Thermo Fisher Scientific, Inc.). Total RNA was reverse-transcribed into cDNA by the application of iScript™ Reverse Transcription Supermix (Bio-Rad Laboratories, Inc.). qPCR was performed with the use of TB Green™ Fast qPCR mix (Takara Bio, Inc.) under the following thermocycling conditions: 95°C for 5 min, followed by 40 cycles at 95°C for 5 sec and 61°C for 30 sec. The primers used for qPCR were presented in **Supplementary Table 2**. Relative mRNA levels were calculated by the 2^-ΔΔCq^ method and normalized to the internal reference gene GAPDH (15).

### CCK-8 Assay and AV/PI Assay

Cell proliferation was detected by CCK-8 assay as follows: A total of 10 μl CCK-8 solution and 90 μl RPMI-1640 mediums were added to the cells in each well and incubated at 37°C with 5% CO_2._ Cell proliferation was measured at 0, 24, 48 and 72 h post-transfection using a microplate reader to determine the optical density value.

Cell apoptosis rate was detected by the AV/PI assay as follows: Cells were digested with pancreatin, washed with PBS and suspended in 100 μl binding buffer. The cells were subsequently incubated with 5 μl AV and 5 μl PI for 15 min at room temperature in the dark. Apoptotic cells were subsequently analyzed using a flow cytometer with Flow Jo software (version 7.6.5, BD, USA).

### Wound Healing Assay and Transwell Assay

Cell migration was detected by the wound healing assay as follows: Cells were cultured until 80% confluence was reached, and a sterile pipette tip was used to introduce a wound, which was set as 0 h. The cells were washed with PBS and incubated at 37°C and 5% CO_2_. The wound was observed using a microscope at 0 and 24 h. The migration rate (ranging from 0-100%) was calculated by dividing the width of the gap at 24 h by that at 0 h.

Cell invasion was detected by the Transwel assay as follows: Transwell chambers (Coring, Inc.; 8-μm pore size; 6.5-mm) were precoated with Matrigel (BD Biosciences) for 2 h at 37°C. The transfected cells were subsequently seeded in the top compartment of the Transwell chambers and incubated at 37°C for 24 hs. Cells on the upper surface were removed and invading cells on the lower surface were fixed using methyl aldehyde (Sigma-Aldrich; Merck KGaA), and then stained with 0.5% crystal violet (Sigma-Aldrich; Merck KGaA) for 15 mins. The number of invading cells in each well was determined by counting the cells in 5 fields of view per well (magnification, x100), subsequently the mean value was assessed.

### Sphere Formation Assay

Stably transfected SKOV3 and OVCAR3 cells were cultured in DMEM/F12 Medium (Gibco; Thermo Fisher Scientific, Inc.) supplemented with 2% B27 (Gibco, Thermo Fisher Scientific, Inc.), 20 ng/ml EGF (Sigma-Aldrich; Merck KGaA), 20 ng/ml bFGF (Gibco; Thermo Fisher Scientific, Inc.) and 4 μg/ml heparin (Sigma-Aldrich; Merck KGaA) for 10 days. The number of spheres with a diameter of >50 μm was counted under a microscope. The sphere formation ability was calculated as: Number of spheres/total number of seeded cells x 1000/1000.

### Patients, Samples and Data Collection

A total of 76 patients with EOC who underwent surgery at the Harbin Medical University Cancer Hospital from January 2013 to December 2017 were retrospectively reviewed in the present study. The inclusion criteria were as follows: i) Histopathologically-confirmed primary EOC diagnosis; ii) >18 years of age; iii) received ovarian cancer resection; iv) availability of complete clinical and pathological data prior to surgery; v) complete OS data; and vi) availability of tumor and paired adjacent tissues stored in liquid nitrogen at the Specimen Storehouse of Harbin Medical University Cancer Hospital. The present study was approved by the Institutional Review Board of Harbin Medical University Cancer Hospital, and written informed consent was obtained from all the patients or their guardians.

Data on patient age, histological subtype, pathological grade, peritoneal cytology, tumor size, volume of ascites, International Federation of Gynecology and Obstetrics (FIGO) stage and carbohydrate antigen 125 levels were retrieved from the Electronic Medical Record System of the Harbin Medical University Cancer Hospital. The OS was calculated from the date of surgery to the date of mortality. The median follow-up duration was 29.0 months (25^th^-75^th^ quintiles, 19.5-44.5 months), and the last follow-up date was 2017/12/31. EOC tumor and adjacent tissue samples were obtained from the Specimen Storehouse of the Harbin Medical University Cancer Hospital, and lnc-TCF7 expression in samples was determined by RT-qPCR.

### Immunohistochemistry (IHC) Assessment

The tumor and adjacent tissue specimens were formalin-fixed, paraffin-embedded and cut into 4-μm thick sections. After the sections were deparaffinized and rehydrated, antigen retrieval was performed by heating in a microwave. Endogenous peroxidase activity was blocked with 0.3% H_2_O_2_ and the sections were subsequently incubated with 10% normal goat serum (Sigma-Aldrich; Merck KGaA) to prevent non-specific binding. Subsequently, the sections were incubated with a rabbit anti-ITGB8 antibody (1:500, ab80673; Abcam) overnight at 4°C. Following primary antibody incubation, the sections were incubated with a horseradish peroxidase-conjugated goat-anti-rabbit secondary antibody (1:1,000, ab205718; Abcam) for 60 min at 37°C. After staining, counterstaining and sealing, the sections were observed under a Nikon ECLIPSE E200 microscope (Nikon Corporation). Staining was assessed by a semi-quantitative scoring method as previously described (16). The total IHC score ranged between 0 and 12, and all tissues were classified as ITGB8 high expression (total IHC score >3) and ITGB8 low expression (total IHC score ≤3).

### Statistical Analysis

Statistical analyses were performed using SPSS software (version 22.0; IBM Corp.) and graphs were drawn using GraphPad software (version 6.01; GraphPad Software, Inc.). Data were presented as the mean ± standard deviation (SD) or median (25^th^-75^th^ quintiles). Comparison between the two groups was performed by the Student’s t-test, Wilcoxon rank sum test or Wilcoxon signed rank sum test, as applicable. Multiple comparisons were determined by one-way analysis of variance (ANOVA) followed by Dunnett’s multiple comparisons test. Survival curves were drawn using the Kaplan-Meier method and compared by the log-rank test. P<0.05 was considered to indicate a statistically significant difference.

## Results

### Effect of lnc-TCF7 Dysregulation on SKOV3 Cell Viability and Mobility

Lnc-TCF7 was increased in EOC cell lines compared to control cell line (**Figure 1A**). In SKOV3 cells, lnc-TCF7 overexpression enhanced cell proliferation, Bcl-2 expression, cell migration and cell invasion, while reduced cell apoptosis, C-Caspase 3 expression (All P<0.05, **Figures 1B–J**). Besides, lnc-TCF7 knockdown exhibited the opposite effect compared to its overexpression (**Figures 1B–J**).

**Figure 1:** Effect of lnc-TCF7 on cell proliferation, apoptosis, migration and invasion in SKOV3 cells. **(A)** The expression of lnc-TCF7 in EOC cells lines and normal ovarian epithelial cells; **(B)** The expression of lnc-TCF7 expression after transfection; **(C)** Cells proliferation in SKOV3 cells; **(D, E)** Cells apoptosis in SKOV3 cells. **(F)** Western blot; **(G, H)** Cells migration in SKOV3 cells; **(I, J)** Cells invasion in SKOV3 cells. Experiments were performed in triplicates. * represented *P* < 0.05, ** represented *P* < 0.01, *** represented *P* < 0.001.

### Effect of lnc-TCF7 Dysregulation on SKOV3 Cell Stemness and Cisplatin Sensitivity

Lnc-TCF7 overexpression promoted CD44 expression, CD133 expression, CD44^+^CD133^+^ cell proportion, sphere formation ability, while decreased cisplatin sensitivity in SKOV3 cells (All P<0.05, **Figures 2A–H**). Besides, lnc-TCF7 knockdown showed the opposite effect compared with its overexpression (**Figures 2A–H**).

**Figure 2:** Effect of lnc-TCF7 on cell stemness in SKOV3 cells. **(A, C)** CD44 expression after transfection; **(B, C)** CD133 expression after transfection; **(D, E)** CD44^+^CD133^+^cell percentage after transfection; **(F, G)** spheres formation efficiency after transfection; **(H)** drug resistance to cisplatin after transfection. Experiments were performed in triplicates. * represented *P* < 0.05, ** represented *P* < 0.01.

### Microarray Analysis and Targets Sorting

Microarray analysis of mRNA profile between the OE-TCF7 and the OE-NC group was performed: Volcano analysis showed the overall mRNA expression pattern between the two groups (**Figure 3A**), then the GO and KEGG enrichments revealed that the DEGs were mainly related to carcinogenetic processes and pathways (**Figures 3B, C** **)**. Besides, microarray analysis of mRNA profile between the SH-TCF7 and the SH-NC group was also carried out: Volcano analysis showed the overall mRNA expression pattern between the two groups (**Figure 3D**), then GO and KEGG enrichments revealed that the DEGs were also linked with carcinogenetic processes and pathways (**Figures 3E, F** **)**.

**Figure 3:** Microarray analysis. Volcano plots **(A)**, GO enrichment **(B)**, KEGG enrichment **(C)** of mRNA profile between OE-TCF7 group vs. OE-NC group; Volcano plots **(D)**, GO enrichment **(E)**, KEGG enrichment **(F)** of mRNA profile between SH-TCF7 group vs. SH-NC group; Cross analysis **(G)**, Heatmap **(H)**, GO enrichment **(I)**, KEGG enrichment **(J)** of accordant mRNA profile.

In addition, cross-analysis was performed to identify the overlapping DEGs between the OE-TCF7 vs. OE-NC groups, between the SH-TCF7 vs. SH-NC groups (**Figures 3G, H** **)**, which were mainly enriched in key oncogene biological processes and pathways (**Figures 3I, J** **)**. Then the information of the top 20 accordant DEGs was listed in **Supplementary Table 3**.

Subsequently, the top 5 according DEGs were chosen as candidate targets, then further validated by western blot and RT-qPCR, respectively (**Figures 4A–F**). The data observed that lnc-TCF7 overexpression increased PCDHB8 expression, ITGB8 expression and decreased FN1 expression, but did not affect SNX2 or IL1A expression. Meanwhile, lnc-TCF7 knockdown reduced ITGB8 expression while elevated IL1A expression, but did not affect SNX2, PCDHB8 or FN1 expression. Collectively, ITGB8 was the most dysregulated one by lnc-TCF7 dysregulation. Therefore, it was chosen for further experiments.

**Figure 4:** Validation of top 5 DEGs expressions after transfection. SNX2 **(A)**, PCDHB8 **(B)**, ITGB8 **(C)**, IL1A **(D)**, FN1 **(E)** mRNA expressions after transfection; and their protein expressions after transfection **(F)**. Experiments were performed in triplicates. * represented *P* < 0.05, ** represented *P* < 0.01, *** represented *P* < 0.001, ns represented no significance.

### Effect of ITGB8 on SKOV3 Cell Viability, Mobility, Stemness and Cisplatin Sensitivity, as well as Its Interaction With lnc-TCF7

ITGB8 overexpression increased cell proliferation, Bcl-2 expression, cell migration, cell invasion, CD133 expression, CD44^+^CD133^+^ cell proportion, sphere formation ability, while decreased cell apoptosis and C-Caspase 3 expression without affecting lnc-TCF7 expression, CD44 expression and cisplatin sensitivity in SKOV3 cells (**Figures 5A–K** and **Figures 6A–F**). Furthermore, ITGB8 overexpression attenuated the effect of lnc-TCF7 knockdown on regulating these cell functions (**Figures 5A–K** and **Figures 6A–F**).

**Figure 5:** Effect of ITGB8 overexpression on cell proliferation, apoptosis, migration and invasion in SKOV3 cells. Lnc-TCF7 expression **(A)**, ITGB8 expression **(B, C)**, cell proliferation **(D)**, cell apoptosis rate and apoptotic markers **(E–G)**, cell migration **(H, I)**, cell invasion **(J, K)** after corresponding transfections. Experiments were performed in triplicates. * represented *P* < 0.05, ** represented *P* < 0.01, *** represented *P* < 0.001, ns represented no significance.

**Figure 6:** Effect of ITGB8 overexpression on cell stemness and cisplatin sensitivity in SKOV3 cells. CD44 **(A)**, CD133 **(B)** mRNA expressions, their protein expressions **(C)**, CD44^+^CD133^+^cell percentage **(D)**, spheres formation efficiency **(E)** and cisplatin sensitivity **(F)** after corresponding transfections. Experiments were performed in triplicates. * represented *P* < 0.05, ** represented *P* < 0.01, ns represented no significance.

### Validation of the Effects of lnc-TCF7 and ITGB8 on Regulating OVCAR3 Cell Functions

In OVCAR3 cells, lnc-TCF7 overexpression enhanced cell proliferation, cell migration, cell invasion, CD44 expression, CD133 expression, CD44^+^CD133^+^ cell proportion, sphere formation ability, but reduced cell apoptosis and cisplatin sensitivity (**Figures 7A–O**). Furthermore, lnc-TCF7 knockdown disclosed opposite effects to its overexpression in OVCAR3 cells (**Figures 7A–O**).

**Figure 7:** Effect of lnc-TCF7 on cell proliferation, apoptosis, migration, invasion, stemness and cisplatin sensitivity in OVCAR3 cells. Lnc-TCF7 expression **(A)**, cell proliferation **(B)**, cell apoptosis rate **(C, D)**, cell migration **(E, F)**, cell invasion **(G, H)**, CD44 expression **(I)**, CD133 expression **(J)** CD44^+^CD133^+^ cell percentage **(K, L)**, spheres formation efficiency **(M, N)** and cisplatin sensitivity **(O)** after corresponding transfections. Experiments were performed in triplicates. * represented *P* < 0.05, ** represented *P* < 0.01, *** represented *P* < 0.001, ns represented no significance.

ITGB8 knockdown descended cell proliferation, cell migration, cell invasion, CD44 expression, CD133 expression, CD44^+^CD133^+^ cell proportion, sphere formation ability, but raised cell apoptosis and cisplatin sensitivity in OVCAR3 cells (**Figures 8A–N**). Furthermore, ITGB8 knockdown alleviated the effect of lnc-TCF7 overexpression on modulating these cell functions (**Figures 8A–N**).

**Figure 8:** Effect of ITGB8 knockdown on cell proliferation, apoptosis, migration, invasion, stemness and cisplatin sensitivity in OVCAR3 cells. Lnc-TCF7 expression **(A)**, ITGB8 expression **(B)**, cell proliferation **(C)**, cell apoptosis rate **(D, E)**, cell migration **(F, G)**, cell invasion **(H, I)**, CD44 expression **(J)**, CD133 expression **(K)** CD44^+^CD133^+^ cell percentage **(L)**, spheres formation efficiency **(M)** and cisplatin sensitivity **(N)** after corresponding transfections. Experiments were performed in triplicates. * represented *P* < 0.05, ** represented *P* < 0.01, *** represented *P* < 0.001, ns represented no significance.

### Lnc-TCF7 and ITGB8 Expressions in EOC Patients

Lnc-TCF7 was upregulated in tumor tissue than in adjacent tissue (P<0.001, **Figure 9A**); meanwhile, it was correlated with higher pathological grade, larger tumor size, and more advanced FIGO stage (all P<0.05, **Table 1**) in EOC patients. Besides, lnc-TCF7 high expression predicted worse OS in EOC patients (P<0.05, **Figure 9B**). Furthermore, lnc-TCF7 positively correlated with ITGB8 expression in EOC tumor tissue, and the latter expression also related to more advanced FIGO stage (all P<0.05, **Figures 9C–G**).

**Figure 9:** Correlation of lnc-TCF7 with ITGB8 and survival. The expression of lnc-TCF7 in tumor tissue and adjacent tissue of EOC **(A)**; The correlation of lnc-TCF7 with OS in EOC patients **(B)**; The correlation of lnc-TCF7 with ITGB8 expression in EOC tumor tissue **(C–E)**; The correlation of ITGB8 with FIGO stage **(F, G)**.

**Table 1:** Correlation of Lnc-TCF7 expression with clinicopathological features.

	Lnc-TCF7 expression	*P* value
Age		0.171
<50years (n=26)	1.760 (1.094-3.665)	
>=50years (n=50)	2.460 (1.775-4.229)	
Histological subtype		0.584
Serous (n=49)	2.450 (1.422-4.640)	
Others (n=27)	2.237 (1.406-4.001)	
Pathological grade		0.028
G1-G2 (n=34)	1.817 (1.318-3.104)	
G3 (n=42)	3.062 (1.904-4.711)	
Peritoneal cytology		0.797
Negative (n=27)	2.149 (1.638-3.148)	
Positive (n=36)	2.413 (1.371-4.537)	
Tumor size		0.014
<10cm (n=37)	1.859 (1.358-3.894)	
>=10cm (n=39)	2.777 (1.782-4.976)	
The volume of ascites		0.105
<100ml (n=26)	1.860 (1.356-3.036)	
>=100ml (n=50)	2.450 (1.546-4.782)	
FIGO stage		<0.001
I-II (n=25)	1.376 (1.086-1.956)	
III-IV (n=51)	3.062 (1.979-5.060)	
CA125		0.204
<1000U/ml (n=51)	2.413 (1.368-3.678)	
>=1000U/ml (n=25)	2.308 (1.546-4.782)	

Data were presented as median (25^th^-75^th^). Comparison between two groups was determined by Wilcoxon rank sum test. P < 0.05 was considered significant. FIGO, International Federation of Gynecology and Obstetrics; CA125, Carbohydrate antigen 125.

## Discussion

EOC is one of the most common causes of mortality among gynecologic malignancies, and a complex disease related to genetic mutations, chromosomal translocations, deletions, amplification or epigenetic alterations (17). The current treatments for EOC, including tumor resection surgery, tumor debulking or chemotherapy have been applied according to different disease stages and individual conditions (17, 18), which has improved the prognosis of patients with EOC. Patients diagnosed at the early stages have a 5-year survival rate of more than 70%, however, patients diagnosed as an advanced stage have a worse prognosis (19–21). Therefore, it is necessary to find out additional effective treatment modalities to improve the prognosis of patients with EOC. Comprehensive understanding and exploration of the molecular mechanisms of tumorigenesis would be beneficial for the development of novel potential drugs, and the identification of biological molecules may help detect cancer in the earlier stages to distinguish different disease subtypes or monitor treatment responses (17, 20).

lncRNAs are emerging as crucial regulators in a variety of biological processes, and have been identified to regulate tumorigenesis through diverse mechanisms, including cotranscriptional regulation, modulation of gene expression, scaffolding of nuclear or cytoplasmic complexes and pairing with other RNAs (22–24). A recent experiment illustrated that lncRNA taurine-upregulated gene 1 mediates aurora kinase A to induce the proliferation and decrease the apoptosis of SKOV3 cells (25). Furthermore, lncRNA sorafenib resistance in renal cell carcinoma associated (LNCSRLR) interacts with Hu antigen R to increase β-catenin expression, which subsequently activates the Wnt/β-catenin signaling pathway to promote cell proliferation. Furthermore, LNCSRLR binds with the miR-200 family to upregulate the expression of zinc finger Ebox binding homeobox (ZEB) 1 and ZEB2 which facilitate the epithelial-mesenchymal transition (EMT), thereby increasing cell invasion in EOC (26). The aforementioned studies illustrated that several lncRNAs play essential roles in the pathology of EOC. However, while over 30,000 lncRNAs have been documented to date, the underlying mechanisms of the majority of these lncRNAs in EOC remain unknown.

lnc-TCF7, one of the most significant cancer-related lncRNAs, is implicated in tumor progression and the regulation of CSC properties by targeting multiple genes and signaling pathways. For example, lnc-TCF7 induced by the IL-6/STAT signaling pathway increases EMT to elevate the aggressiveness of hepatocellular carcinoma (8, 27). Additionally, lnc-TCF7 facilitates the self-renewal ability of CSCs *via* the activation of the Wnt signaling pathway by recruiting the switch/sucrose non-fermentable (SWI/SNF) complex for the upregulation of TCF7 in liver cancer (9). TCF7, a member of the T-cell factor family of transcription factors, is well known for its role in the development of T lymphocytes, which are related to tumorigenesis and tumor progression (28). According to previous studies, the N-terminal portion of TCF7 contains the β-catenin-binding domain that is important for Wnt signaling-determined tumorigenicity, which suggests that TCF7 may act as a Wnt effector in carcinomas (29, 30). The SWI/SNF complex is known as an evolutionarily-conserved multisubunit chromatin-remodeling complex, and Brg1/Brm-associated factor 170 (BAF170) is an SWI/SNF-related, matrix-associated, actin-dependent regulator of chromatin subfamily c member. Growing evidence indicates that the levels of SWI/SNF subunits may be regulated by BAF170 (31). The studies mentioned above suggested that lnc-TCF7 may bind to BAF170 and influence BAF170 binding to the -1,200 to -1,100 bp segment of the TCF7 promoter to promote self-renewal of human liver CSCs (9, 31). Therefore, TCF7 is a key transcription factor that promotes the self-renewal ability of cancer cells in different carcinomas. Furthermore, lnc-TCF7 may function as an oncogene by inducing CSC properties by regulating the expression of TCF7. lnc-TCF7 possesses a potential function as a tumor promoter by increasing aggressiveness or CSC properties in several types of cancer.

lnc-TCF7 silencing was found to inhibit the proliferation, migration and invasion of the colorectal cancer cell lines SW-620 and HT29 (12). Lnc-TCF7 silencing reduced cell migration and invasion by inhibiting TCF7 expression (10). Another *in vitro* experiment revealed that knockdown of lnc-TCF7 decreased cell invasion in the hepatocellular carcinoma cells line SK-Hep-1 (8). Furthermore, lnc-TCF7 overexpression increased cell invasion, while lnc-TCF7 silencing by shRNA decreased cells invasion in the NSCLC cell lines A549 and 95D (7). Therefore, the studies as mentioned earlier suggested that lnc-TCF7 may serve as a tumor promoter in several carcinomas. In order to investigate whether lnc-TCF7 affected cell function in EOC, five common EOC cells lines including CAOV3, SKOV3, OVCAR3 and UWB1.289, were investigated in the present study. The results elucidated that lnc-TCF7 expression was increased in these five EOC cell lines compared with normal cells. The highest and lowest lnc-TCF7 expression levels were observed in SKOV3 and OVCAR3 cells, respectively, compared with IOSE80 cells. Therefore, SKOV3 and OVCAR3 cells were selected for the subsequent experimentation, which found that lnc-TCF7 promoted the proliferation, migration and invasion, but inhibited the apoptosis of SKOV3 and OVCAR3 cells. Therefore, it is suggested that lnc-TCF7 might be a potential therapeutic target in EOC. In clinical samples, the median value of lnc-TCF7 expression in adjacent tissue was 1, and lnc-TCF7 expression ranged from 0.848 to 9.462 in tumor tissue, with a median value of 2.1 times higher than what was observed in adjacent tissue. In EOC cell lines, the median value of lnc-TCF7 expression was 2-3 times exceeding what was observed in the normal ovarian epithelial cell line. The results suggested more variability in lnc-TCF7 expression in the tumor tissue, indicating a higher heterogeneity. However, the trend of increased lnc-TCF7 expression was consistent in both the EOC clinical samples and cell lines.

Furthermore, the effect of lnc-TCF7 on the regulation of cancer cell stemness was investigated in the present study by determining the expression levels of common CSC markers (CD44 and CD133), the CD44^+^CD133^+^ cell proportion, sphere formation ability and drug resistance to cisplatin. CSCs are defined as specific cells within the tumor cell mass that retain a self-renewing ability, and are resistant to chemotherapy or radiotherapy. Furthermore, CSCs have been shown to participate in tumor development, metastasis and recurrence (32). There are several cell surface markers frequently used to identify CSCs in EOC, including CD44 and CD133 (33–35). In the present study, lnc-TCF7 promoted the expression of CD44 and CD133, enhanced the CD44^+^CD133^+^ cell proportion, increased the sphere formation ability and increased drug resistance to cisplatin in SKOV3 and OVCAR3 cells. These findings suggested that lnc-TCF7 may play an important role in priming the CSC properties in EOC. The possible explanation was that: lnc-TCF7 mediated CSC-related pathways (such as promoting Wnt signaling) to induce CSC properties (such as self-renewal ability) in EOC.

In order to explore how lnc-TCF7 regulated cancer cell function and stemness, a microarray analysis of mRNA expression profiles affected by lnc-TCF7 regulation was performed. This revealed that 212 DEGs were upregulated and downregulated in the OE-TCF7 and SH-TCF7 groups, respectively, and 55 DEGs were downregulated and upregulated in the OE-TCF7 and SH-TCF7 groups, respectively. Subsequently, enrichment analysis was performed to identify the biological processes involved in the DEGs induced by lnc-TCF7 dysregulation. The results showed that the consistent DEGs were enriched in a number of biological processes and disease pathways, such as ‘pathways in cancer’, ‘renal cell carcinoma’, ‘choline metabolism in cancer’ and ‘melanoma’. Cancer-associated pathways are involved in the promotion of cell proliferation, migration and invasion, thereby contributing to the processes of tumorigenesis and tumor development in several carcinomas (including colorectal carcinoma, lung cancer and papillary thyroid cancer) (36–38). Renal cell carcinoma is closely related to the sustained growth of the tumor and highly invasive molecules, similarly to EOC (39). Choline metabolism in cancer has been reported to increase phosphocholine and total choline-containing compounds, which may be used to monitor morphological and metabolic changes in the tumor (40). In melanoma, several genes and pathways that promote tumor development may also be relevant to EOC (41).

A total of five candidate genes (including SNX2, PCDHB8, ITGB8, IL-1A and FN1) that are regulated by lnc-TCF7 in EOC were selected according to the rank of the sum of absolute value of Log_2_FC [OE-TCF7 vs. OE-NC] and Log_2_FC [SH-TCF7 vs. SH-NC] in the microarray analysis. RT-qPCR assays revealed that lnc-TCF7 upregulation increased ITGB8 expression, while lnc-TCF7 silencing decreased ITGB8 expression in EOC cells. In order to investigate whether lnc-TCF7 regulated EOC cell functions by upregulating ITGB8, compensational experiments were performed. ITGB8, a member of the integrin β-chain family (ITGB8, Gene ID: 3696; Location: 7p21.1, GRCh38.p13 NC_000007.14 (20329819…20415754); transcript ID: NM_002214.3.), has been reported to be highly expressed in a variety of malignant tumors, such as laryngeal squamous cell carcinoma, and is therefore a key metastasis-related gene and a potential therapeutic target (42, 43). Furthermore, ITGB8 may interact with different genes or pathways to promote tumorigenesis. For example, ITGB8 interacts with miR19b-3p to induce cell proliferation, migration and invasion, which accelerate tumor growth and metastasis in colorectal cancer (44). ITGB8 silencing inhibits Snail and nuclear factor κB transcriptional activity, thereby decreasing the metastatic potential in the human lung cancer cell lines A549 and PC9 (42). Another *in vitro* experiment revealed that ITGB8 promoted gefitinib resistance in hepatic cancer, facilitated the cell cycle and decreased cell apoptosis by interacting with the transforming growth factor β pathway in the HepG2/G cell line (45). In ovarian cancer, ITGB8 overexpression enhanced cisplatin resistance in SKOV3 cells (46). Therefore, the aforementioned studies suggested that ITGB8 may influence cellular activities or drug sensitivity by mediating various genes or pathways. The present study revealed that lnc-TCF7 was likely to regulate cellular functions and stemness in EOC by upregulating ITGB8. Further compensational experiments were performed to validate this hypothesis and disclosed that lnc-TCF7 increased the proliferation, migration, invasion and stemness but decreased apoptosis of EOC cells by upregulating ITGB8. These data further demonstrated the role of lnc-TCF7 in the etiology of EOC and potential therapeutic targets.

LncRNAs serve as competitive endogenous RNAs by competitively binding with miRNAs to regulate targeted mRNAs (47, 48). Therefore, lnc-TCF7 may regulate ITGB8 by interacting with various upstream miRNAs in EOC cells. The present study was performed to detect the target genes of lnc-TCF7, and then screened out the possibility of the regulatory relationships between lnc-TCF7 and ITGB8. Whereas the library process of miRNA sequencing differed a lot compared to mRNA sequencing, and miRNA expression profile was not detected in our study. Therefore, while an association between lnc-TCF7 and ITGB8 in EOC cells was established, the direct or indirect effects of lnc-TCF7 on ITGB8 remain unclear. Based on previous evidence, lnc-TCF7 may mediate the function of several miRNAs (including miR-200c, miR-92a, miR-135b), and these miRNAs may also regulate ITGB8 (predicted by RNAHybrid, PITA and miRanda databases) (49). However, related miRNAs were not investigated in the present study. Therefore, future studies investigating the roles of miRNAs are required to enhance our understanding of the underlying mechanisms of EOC. Additionally, the effect of lnc-TCF7 on cellular function in normal cell lines was not performed in the study, and this should be explored in future studies. What’s more, lack of animal studies for validation was still the main limitation in this study. Hence, further animal study was needed.

Lnc-TCF7 is highly expressed in different carcinomas, including colorectal cancer, hepatocellular carcinoma and non-small cell lung cancer (7, 9, 12). To the best of our knowledge, only one clinical study has shown that high expression of lnc-TCF7 is correlated with larger tumor size, poor differentiation degree, increased TNM grade, more advanced lymph node metastasis and deeper invasion in patients with colorectal cancer (12). These results suggested that lnc-TCF7 may be upregulated in different types of cancer and may be correlated with clinicopathological features. However, little is known about the correlation of lnc-TCF7 with clinicopathological features in patients with EOC. The present study investigated 76 patients with EOC who underwent surgery and suggested that lnc-TCF7 expression was increased in tumor tissue compared with adjacent tissue. Furthermore, increased lnc-TCF7 expression was associated with higher pathological grade, larger tumor size and FIGO stage in patients with EOC. These observations may be caused by a number of the following reasons. Firstly, lnc-TCF7 accelerated tumor growth and metastasis by promoting EMT, thus it was associated with larger tumor size and more advanced FIGO stage. Secondly, lnc-TCF7 induced CSC properties (such as self-renewal ability) by regulating related pathways (such as facilitating the Wnt signaling pathway), consequently leading to increased pathological grade in patients with EOC. Thirdly, the microarray analysis of mRNA expression profiles in the present study revealed that lnc-TCF7 was mainly implicated in regulating cancer-related genes and pathways in EOC, which contributes to the increased pathological grade, larger tumor size and advanced FIGO stage. The present study also revealed that high expression of lnc-TCF7 was associated with a shorter OS in patients with EOC, which could be explained by that: Firstly, lnc-TCF7 was associated with advanced disease stage in patients with EOC, which indirectly resulted in poor prognosis. Secondly, lnc-TCF7 promoted EOC cells stemness to increase drug resistance and metastasis risk, thereby causing a worse prognosis in patients with EOC. Thirdly, according to the results of microarray analysis in the present study, lnc-TCF7 may regulate cancer-related genes and pathways to accelerate tumor progression, thus leading to a poor prognosis in patients with EOC. These results suggested that lnc-TCF7 may act as a novel biomarker for tumor progression and prognosis in patients with EOC.

Several limitations existed in this study: (1) The NC group but not blank control group was set in the current study, which needed further validation; (2) The mechanism between lnc-TCF7/ITGB8 network and potentially regulated pathways in EOC could be explored in the future studies; (3) The lnc-TCF7 in EOC cells was investigated in the current study, while its effect in normal cell lines was still obscure, which could be further exploration; (4) lacking *in vivo* experiment was an important limitation of our study, which should be assessed in our following studies; (5) In the clinical part of our study, the sample size of EOC patients was relatively small, therefore, further validation in a larger patient cohorts was required; (6) The clinical part of our study retrospectively analyzed EOC patients from a single center, therefore, a multi-center, prospective study was needed in the future; (7) The lnc-TCF7 and ITGB8 expressions was detected in tumor tissue and adjacent tissue of EOC patients, while their expressions in normal ovarian tissue needed further detection.

To be conclusive, lnc-TCF7 not only promotes EOC viability, mobility and stemness *via* regulating ITGB8, but also correlates with worse tumor features and survival in EOC patients. These imply its potency as a target for EOC treatment.

## Data Availability Statement

The original contributions presented in the study are included in the article/**Supplementary Material**. Further inquiries can be directed to the corresponding author.

## Ethics Statement

The studies involving human participants were reviewed and approved by Institutional Review Board of Harbin Medical University Cancer Hospital. The patients/participants provided their written informed consent to participate in this study.

## Author Contributions

KH contributed conception and design of the study. CS performed the statistical analysis and wrote the first draft of the manuscript. CS contributed to data acquisition. KH contributed to manuscript revision. All authors contributed to data interpretation and approved the final version.

## Funding

This study was supported by BeiJing Heart To Heart Foundation (HXXT2021ktyj002), Beijing Medical Award Foundation (YXJL-2021-0763-0482), and Beijing Medical Award Foundation (YXJL-2021-0508-0378).

## Conflict of Interest

The authors declare that the research was conducted in the absence of any commercial or financial relationships that could be construed as a potential conflict of interest.

## Publisher’s Note

All claims expressed in this article are solely those of the authors and do not necessarily represent those of their affiliated organizations, or those of the publisher, the editors and the reviewers. Any product that may be evaluated in this article, or claim that may be made by its manufacturer, is not guaranteed or endorsed by the publisher.
